# Modified Immune Evolutionary Algorithm for Medical Data Clustering and Feature Extraction under Cloud Computing Environment

**DOI:** 10.1155/2020/1051394

**Published:** 2020-01-20

**Authors:** Jing Yu, Hang Li, Desheng Liu

**Affiliations:** ^1^Luxun Academy of Fine Arts, No. 19, Miyoshi Street, HePing District, Shenyang P. C 110000, China; ^2^Software College, Shenyang Normal University, Shenyang 110034, China; ^3^College of Information and Electronic Technology, Jiamusi University, Jiamusi 154007, Heilongjiang, China

## Abstract

Medical data have the characteristics of particularity and complexity. Big data clustering plays a significant role in the area of medicine. The traditional clustering algorithms are easily falling into local extreme value. It will generate clustering deviation, and the clustering effect is poor. Therefore, we propose a new medical big data clustering algorithm based on the modified immune evolutionary method under cloud computing environment to overcome the above disadvantages in this paper. Firstly, we analyze the big data structure model under cloud computing environment. Secondly, we give the detailed modified immune evolutionary method to cluster medical data including encoding, constructing fitness function, and selecting genetic operators. Finally, the experiments show that this new approach can improve the accuracy of data classification, reduce the error rate, and improve the performance of data mining and feature extraction for medical data clustering.

## 1. Introduction

Through the support of existing technologies, relevant medical research organizations only rely on coupled dictionary technology to classify and store medical images [1]. However, with the continuous increase of the number of slices, some images begin to show serious frame rate overlap phenomenon, which not only causes the sharp decline of the original image gray level but also causes a series of image data redundancy problems. It brings great trouble to the mining and scheduling of the following image information. The so-called image data redundancy refers to the phenomenon of uneven or excessive storage caused by data repetition in the process of data imaging that can lead to the real information loss in the image and cause a certain negative impact on the image sharpness. Frame rate overlap is a common image fault problem, which is often associated with image data redundancy. Under certain circumstances [2], a certain degree of frame rate overlap may lead to a small increase of the image sharpness. But excessive frame rate overlap will lead to serious damage to the modal property of the medical image, which will lead to a large increase of the redundant region in the medical image data. Diagnosis in medicine is related to the patient's medication and treatment. Many diseases are more complex. Data clustering analysis is integrated into the diagnosis of diseases, such as clinical urology and breast cancer, so that doctors can greatly enhance the diagnosis accuracy of patients.

With the fast growth of information science, the research of biological applications has been used for computational science to analyze the intelligent bionic optimization algorithm design and improve the ability of processing big data and analysis [3]. Intelligent bionic algorithms mainly include ant colony algorithm [4], particle swarm optimization (PSO) algorithm [5], and the quantum swarm algorithm [6–8]. Swarm intelligence optimization algorithms have a good application value in artificial intelligence design, data clustering analysis, computer control, and other fields.

Clustering technology is an important part in data mining and machine learning. Domestic researchers mainly focus on the following two aspects: (1) a clustering algorithm dynamically determines the number of clustering centers and (2) a clustering algorithm improves the accuracy of clustering. Zhao et al. [9] presented a new dynamic clustering method based on genetic algorithm; the main idea of the method was that, in order to effectively overcome the sensitivity to the initial state value clustering algorithm, it used the maximum attribute value range partitioning strategy and two stages and dynamic selection method in mutation, which obtained the optimal clustering center.

Clustering analysis is a kind of unsupervised model in pattern recognition. The task of cluster is to divide an unmarked pattern according to the certain criteria into several subsets, which requires that similar samples have the most similar cluster center and dissimilar samples should be divided in different classes. Therefore, it is also called unsupervised classification. Clustering analysis has been extensively used in data mining, image processing, object detection, radar target detection, etc. [10, 11]. Zhang et al. [12] proposed a Geometric-constrained multiview image matching method based on semiglobal optimization. It was obvious that some features had more information than others in a dataset. So it was highly likely that some features should have lower importance degrees during a clustering or a classification algorithm due to their lower information, their higher variances, etc. So, it was always a desire for all artificial intelligence communities to enforce the weighting mechanism in any task that identically used a number of features to make a decision. Parvin and Minaei-Bidgoli [13] proposed a weighted locally adaptive clustering algorithm that was based on the locally adaptive clustering algorithm.

Nowadays, different clustering methods are being used to resolve several machine learning problems. According to the clustering criterion, different clustering algorithms can be divided into clustering algorithm based on fuzzy relations including hierarchical clustering and graph clustering and clustering algorithm based on the objective function [14–16]. For the objective function of optimization clustering algorithms, it generally uses the gradient method to solve the extremum problem. The search direction of gradient method is always along the direction of the energy reduction, which prompts the algorithm easily falling into local minimum value. Methods are sensitive to the initialization of clustering algorithm in the objective function which is a serious defect. To overcome the above shortcomings, all proposed algorithms are used to optimize objective function. Meng et al. [17] presented that the MapReduce programming model was adopted to combine Canopy and K-means clustering algorithms within cloud computing environment, so as to fully utilize the computing and storing capacity of Hadoop clustering. Large quantities of buyers on taobao were taken as application context to do case study through the Hadoop platform's data mining set Mahout. Zhang et al. [18] proposed a high-order possibilistic c-means algorithm (HOPCM) for big data clustering by optimizing the objective function in the tensor space. Li et al. [19] proposed a task scheduling algorithm based on fuzzy clustering algorithms. However, there are still some problems, such as long convergence time.

Moreover, deep learning-based methods are used for feature selection. Minaei-Bidgoli et al. [20] proposed an ensemble based approach for feature selection. The results showed that, although the efficacy of the method was not considerably decreased in most of cases, the method became free from setting of any parameter. Some algorithms could not properly represent data distribution characteristics when datasets were imbalanced. In some cases, the cost of wrong classification could be very high in a sample of a special class, such as wrongly misclassifying cancerous individuals or patients as healthy ones. Hu and Du [21] tried to present a fast and efficient way to learn from imbalanced data. This method was more suitable for learning from the imbalanced data having very little data in class of minority. Gao et al. [22] was devoted to the exploration of brain images for early detection of Parkinson's disease. All brain images were analyzed to extract Gabor 2D features. It was also shown that the models created on Gabor features outperform the ones created without Gabor features. Zhao et al. [23] analyzed the triple-negative breast neoplasm gene regulatory network using gene expression data. We collected triple-negative breast neoplasm gene expression data from the Cancer Genome Atlas to construct a triple-negative breast neoplasm gene regulatory network using least absolute shrinkage and selection operator regression. In addition, it constructed a triple-positive breast neoplasm network for comparison. Nejatian [24] presented that the available additional information at different times and conditions and gold-standard protein complexes was employed to determine fitting thresholds. By doing so, the problem was converted into an optimization problem. Thereafter, the problem was solved using the firefly metaheuristic optimization algorithm.

Hence, we propose a new medical big data clustering algorithm based on modified immune evolutionary method under cloud computing environment to overcome the above disadvantages in this paper. The reminder of this paper is organized as follows: Section 2 presents big data structure analysis in cloud computing environment. Immune evolutionary algorithm is stated in Section 3.  Section 4 describes the improved clustering method in detail, Section 5 provides the MapReduce framework, and Section 6 manifests the experiments results. Finally, the conclusion is given in Section 7.

## 2. Analysis on Storage Mechanism and Structure of Medical Big Data in Cloud Computing Environment

Cloud computing [25–28] is through the Internet to provide dynamic data to extend large storage space and the structure model. In order to evaluate the data clustering and mining in the cloud computing environment, it needs to build a big data storage system architecture in cloud computing environment. Big data storage structure adopts virtualized storage pool and depends on the computer cluster. From top to bottom, these are the I/O (input/output) virtual computer, USB interface layer sequence, and disk layer, respectively. Enterprise data center through all kinds of terminal accesses the application service, which makes the calculation of distribution on a large number of distributed computers. When all the cloud computing virtual machines are assigned to the physical machine, it uses the following formula to calculate the global optimal solution in this clustering process. And, it also can assign big data feature clustering center BF_M_*i*__ of the cloud computing on the physical machine *P*_M_*i*__ according to the optimal solution:

(1) $$\begin{array}{c} N=\frac{1}{n}\overset{n}{\underset{j=1}{\sum }}\left|U_{t_{j}^{\text{CPU}}}-U_{t_{\text{avg}}^{\text{CPU}}}\right|+\frac{1}{n}\overset{n}{\underset{j=1}{\sum }}\left|U_{t_{j}^{\text{Mem}}}-U_{t_{\text{avg}}^{\text{Mem}}}\right|+\frac{1}{n}\overset{n}{\underset{j=1}{\sum }}\left|U_{t_{j}^{\text{bw}}}-U_{t_{\text{avg}}^{\text{bw}}}\right|. \end{array}$$

The sample is collected and analyzed to determine whether the sample belongs to a typical sample. Assuming that data information stream sample $S=\left({\bar{X}}_{1},{\bar{X}}_{2},\ldots ,{\bar{X}}_{k}\right)$ makes sampling in time (*T*_1_, *T*_2_,…, *T*_*k*_). We divide big data set *X* in cloud environment into *c* clusters, 1 < *c* < *n*. The data segmentation can be transformed as space segmentation. Storage structure central vector of big data is obtained:

(2) $$\begin{array}{c} V=\left\{\left.v_{ij}\right|i=1,2,\ldots ,c,j=1,2,\ldots ,s\right\}, \end{array}$$

where *V*_*i*_ is the *i*-th vector of object cluster feature.

Fuzzy division matrix can be presented as

(3) $$\begin{array}{c} U=\left\{\left.\mu_{ik}\right|i=1,2,\ldots ,c,\;k=1,2,\ldots ,n\right\}. \end{array}$$

Redundant data reduction is processed for a single data source. In the process of multichannel QoS demand virtual machine clustering, some parameters are defined as virtual machine set *V*_MS_={*V*_M_1__, *V*_M_1__,…, *V*_M_m__} and physical machine set *P*_MS_={*P*_M_1__, *P*_M_1__,…, *P*_M_*n*__}. Inspiring factor is *α*, and the expect of inspiring factor is *β*. Biggest mining number is *I*_max_. As a result, uploaded data blocks provide a fixed size of data blocks, which is beneficial to analyze the cloud clustering. Through the big data storage mechanism analysis in cloud computing environment, it provides the accurate data for big data clustering.

Supposing that the time series of information stream is {*x*(*t*_0_+*i*Δ*t*)}, *i*=1,2,…, *N* − 1. *X* and *Y* are attribute sets. The vector expression of big data clustering space in the cloud computing environment is

(4) $$\begin{array}{c} ℜ=\left[r\left(t_{0}\right),r\left(t_{0}+\Delta t\right),\ldots ,r\left(t_{0}+\left(K-1\right)\Delta t\right)\right], \end{array}$$

where *r*(*t*) is information stream time series of big data clustering in cloud computing environment and Δ*t* is data sampling interval. The spectral characteristic *X*_p_(*u*) of discrete samples of big data can be calculated as

(5) $$\begin{array}{c} X_{\text{p}}\left(u\right)=s_{\text{c}}\left(t\right)e^{2\pi f_{0}t}=\frac{1}{\sqrt{T}}\text{rect}\frac{t}{T}e^{\left(2\pi \left(f_{0}t+Kt^{2}\right)/2\right)}, \end{array}$$

where *s*_c_(*t*) is the characteristic scalar time series of big data, *e*^2*πf*_0_*t*^ is the discrete sample center of big data clustering, and (*F*, *Q*) is sample data high-order Bessel function statistics of data set {*X*_1_, *X*_2_,…, *X*_*N*_}. So, we can get the confidence and confidence interval:

(6) $$\begin{array}{c} z_{i,d}^{k+1}=x_{{\text{r}}_{1}}^{k}+F\cdot \left(x_{{\text{r}}_{2}}^{k}-x_{{\text{r}}_{3}}^{k}\right),\\ u_{i,d}^{k+1}=\left\{\begin{array}{c} x_{i\;d}^{t+1},\;f_{\text{fit}}^{t}<f_{\text{fit}}^{\prime },\\ z_{i,d}^{k+1},\;f_{\text{fit}}^{t}\geq f_{\text{fit}}^{\prime }. \end{array}\right. \end{array}$$

Suppose the information flow time series in the cloud computing environment is {*x*(*t*_0_+*i*Δ*t*)}, *i*=0,1,…, *N* − 1. Let *X* and *Y* be the set of properties. The expression of clustering space state vector of big data in cloud computing environment is as follows:

(7) $$\begin{array}{c} X=\left[x\left(t_{0}\right),x\left(t_{0}+\Delta t\right),\ldots ,x\left(t_{0}+\left(K-1\right)\Delta t\right)\right]\\ =\left[\begin{array}{cccc} x\left(t_{0}\right) & x\left(t_{0}+\Delta t\right) & \cdots & x\left(t_{0}+\left(K-1\right)\Delta t\right)\\ x\left(t_{0}+J\Delta t\right) & x\left(t_{0}+\left(J+1\right)\Delta t\right) & \cdots & x\left(t_{0}+\left(K-1\right)\Delta t+J\Delta t\right)\\ \vdots & \vdots & & \vdots \\ x\left(t_{0}+\left(m-1\right)J\Delta t\right) & x\left(t_{0}+\left(1+\left(m-1\right)J\right)\Delta t\right) & \cdots & x\left(t_{0}+\left(N-1\right)\Delta t\right) \end{array}\right], \end{array}$$

where *x*(*t*) is the information flow time series of big data clustering system in cloud computing environment, *J* is the time window function of phase space reconstructed by big data in cloud computing environment, *M* is the target clustering regulator, and Δ*t* is the data sampling interval.

The discrete sample spectral characteristic *X*_p_(*u*) of big data is calculated, and the main feature component is

(8) $$\begin{array}{c} X_{\text{p}}\left(u\right)=s_{\text{c}}\left(t\right)e^{j2\pi f_{0}t}=\frac{1}{\sqrt{T}}\text{rect}\left(\frac{t}{T}\right)e^{j2\pi \left(f_{0}t+Kt^{2}\right)/2}, \end{array}$$

where *s*_c_(*t*) is the characteristic scalar time series of big data and *e*^*j*2*πf*_0_*t*^ is the center of discrete sample of big data clustering.

The data set is {*X*_1_, *X*_2_,…, *X*_*n*_}. (*F*, *Q*) is the high-order Bessel function statistics of the sample data to determine the confidence of node data packets and establish the confidence interval. The obtained confidence and confidence intervals are

(9) $$\begin{array}{c} z_{\left(i,d\right)}^{\left(k+1\right)}=x_{{\text{r}}_{1}}^{k}+F\cdot \left(x_{{\text{r}}_{2}}^{k}-x_{{\text{r}}_{3}}^{k}\right),\\ u_{\left(i,d\right)}^{\left(k+1\right)}=\left\{\begin{array}{cc} x_{id}^{\left(t+1\right)}, & f_{\text{fitness}}^{t}<f_{\text{fitness}}^{*},\\ z_{\left(i,d\right)}^{\left(k+1\right)}, & f_{\text{fitness}}^{t}\geq f_{\text{fitness}}^{*}. \end{array}\right. \end{array}$$

## 3. Immune Evolutionary Algorithm (IEA)

IEA consists of crossover and mutation operator which represent two strategies with group search and information exchange. It provides optimization opportunities for each individual. However, this inevitably produces the degradation phenomenon in some cases, and the degradation phenomenon is quite obvious.

IEA uses some features or knowledge in original problems to suppress the degradation phenomenon appeared in the process of optimization. The key operation of IEA is to construct the structure of immune operator that is finished through vaccination and immune selection. The immune evolutionary algorithm can improve the fitness of the individual and prevent the group degradation, so as to reduce the original wave phenomenon in the late evolutionary algorithm and improve the convergence speed. The main steps for immune evolutionary algorithm are as follows, and the detailed information can be obtained from [29, 30].

1. Randomly generate the initial parent group *A*_1_.
2. Extract the vaccine according to prior knowledge.
3. If the current group contains the best individual, it stops running the process and outputs the result. Otherwise, the procedure continues to work.
4. Cross operation of the current *k*-th group *A*_*k*_ is conducted, and it obtains the population *B*_*k*_.
5. It makes mutation operation for *B*_*k*_ and obtains the population *C*_*k*_.
6. It executes vaccination for *C*_*k*_ and gets group *D*_*k*_.
7. It executes immune selection for *D*_*k*_ and obtains new parent group *A*_*k*+1_. Then back to step 3.

## 4. Modified Immune Evolutionary Algorithm for Data Clustering

Fuzzy clustering is regarded as one of the commonly used approaches for data analysis. The Fuzzy C-means (FCM) algorithm is the most well-known and widely used method for fuzzy clustering and provides an optimal way to construct fuzzy information granules [31]. Cluster prototypes and membership values of data across all clusters can be developed by optimizing the FCM clustering model. Basically, the FCM is a steepest-descent algorithm with variable step length that is adjusted according to the majorization principle for the step length, showing the simplicity and efficiency of the algorithm. Therefore, we combine immune evolutionary algorithm and FCM to optimize the cluster result [32, 33]. The detailed improved data clustering processes are as follows:

The objective function of FCM is

(10) $$\begin{array}{c} J\left(X;U,V\right)=\overset{n}{\underset{k=1}{\sum }}\overset{c}{\underset{i=1}{\sum }}u_{ik}^{m}D_{ik}^{2}, \end{array}$$

(11) $$\begin{array}{c} D_{ik}^{2}={\left(x_{k}-v_{i}\right)}^{T}\left(x_{k}-v_{i}\right), \end{array}$$

where *D*_*ik*_ is the distance from *k*-th data point to *i*-th cluster center, *V*=(*v*_1_, *v*_2_,…, *v*_*c*_) denotes the cluster center of each class, and *v*_*i*_ ∈ *R* and *m* ∈ (1, *∞*) are fuzzy index:

(12) $$\begin{array}{c} X=\left(x_{1},x_{2},\ldots ,x_{n}\right)\subset R,\\ U=\left\{U\in R^{c\times n}\left|u_{ik}\right.\in \left[0,1\right];\overset{c}{\underset{i=1}{\sum }}v_{ik}=1;0<\overset{n}{\underset{k=1}{\sum }}v_{ik}<n\right\}. \end{array}$$

### 4.1. Encoding

According to *J*(*X*; *U*, *V*), the aim of cluster is to obtain fuzzy division matrix *U* and cluster prototype *V* of sample *X*. *U* and *V* are associated with each other. So we have two encoding methods. First, we encode *U*. Suppose that *n* samples need to be divided into *c* clusters. Gene cluster *a*={*α*_1_, *α*_2_,…, *α*_*n*_} denotes one clustering result; *α*_*i*_ ∈ {1,2,…, *c*}. When *α*_*i*_=*k*(1 ≤ *k* ≤ *c*), then *x*_*i*_ belongs to *k*-th cluster. Its search space is *c*^*n*^. If the data samples are bigger, the search space of this encoding is very big too. Therefore, we adopt the second encoding method for *V*. The quantized values are encoded into strings according to their respective values. *a*={*α*_1_, *α*_2_,…, *α*_*l*_}, *l*=*c* × *p*. The former *p* quantized values denote the first *p* dimension cluster center. But it does not change with the data sample *n*.

### 4.2. Constructing Fitness Function

According to *J*(*X*; *U*, *V*), if the clustering effect is better, the object function value is smaller. The formula (10) is used for constructing fitness function *f*:

(13) $$\begin{array}{c} f=\frac{1}{J\left(X;U,V\right)+1}. \end{array}$$

### 4.3. Genetic Operator Selection

Genetic operator has a point crossover, two-point crossover, and multipoint crossover methods. The immune operator inverts the selected individual genes based on certain probability. We can also adopt a reverse genetic mutation operator, namely, it randomly generates a gene in the parent group and the gene is reverted. It basically prevents premature phenomenon. In genetic selection methods, it adopts the roulette wheel selection method and ranking selection. Crossover probability *p*_*c*_ ∈ [0.75, 0.95], *p*_*m*_ ∈ [10^−3^, 10^−2^].

### 4.4. Immune Vaccine Selection

The immune vaccine selection properly describe two ways. It is not clear. Specifically, the first method, after collecting information, executes the immune vaccine. The other is an adaptive method, namely, in the process of group evolution from the best individual genes. It extracts useful information and then executes the vaccine. The former is restricted due to two reasons. The first one is it is difficult to form a mature approach for a prior knowledge. It cannot get effective immune vaccine. The second is, to extract the vaccine, the work costs too much. Therefore, in the clustering algorithm based on immune evolution, we adopt the adaptive method to extract the vaccine.

Therefore, we get the new cluster algorithm as follows (Figure 1).

*Step 1*. Fix cluster class number *c*, 1 ≤ *c* ≤ *n* − 1. Set fuzzy index *m* ∈ (1, +*∞*), stop condition *τ*, total population number *p*_*n*_, crossover probability *p*_*c*_, mutation probability *p*_*m*_, vaccination probability *p*_*v*_, and vaccine update probability *p*_*u*_.
*Step 2*. Randomly generate group *P*(*k*) with *p*_*n*_ individuals.
*Step 3*. Compute fitness of every individual.
  1. Each individual is decoded to calculate each prototype parameter *v*_*i*_, 1 ≤ *i* ≤ *c*.
  2. Use *v*_*i*_ and (8) to calculate *D*_*ik*_^2^.
  3. Calculate *U*=[*u*_*ik*_]_*c*×*n*_.
  4. If *I*_*k*_=*φ*,

(14) $$\begin{array}{c} u_{ik}=\frac{1}{\sum_{j=1}^{c}{\left[d_{ik}^{2}/d_{jk}^{2}\right]}^{\left(1/\left(m-1\right)\right)}}. \end{array}$$

  If *I*_*k*_ ≠ *φ*,

(15) $$\begin{array}{c} u_{ik}=0,\;\forall i\in^{-}I_{k},\\ \underset{i\in I_{k}}{\sum }u_{ik}=1, \end{array}$$

  where *I*_*k*_={*i*|1 ≤ *i* ≤ *c*, *d*_*ik*_=0} and ^−^*I*_*k*_={1,2,…, *c*} − *I*_*k*_.

(4) Use *U*, *D*_*ik*_, and (7) to calculate object function *J*(*X*; *U*, *V*), and then it can get *f* for each individual.

 
*Step 4*. Make statistics for parent group, determine the best individual, then decompose the best individual, and extract immune vaccine *H*={*h*_*i*_|*i*=1 − *m*}.

 
*Step 5*. Use *p*_*c*_ and *p*_*m*_ to make crossover, mutation operation for *P*(*k*), and get group *P*′(*k*).

 
*Step 6*. Execute vaccination and immunization selection for *P*(*k*) and get group *P*(*k*+1).

 
*Step 7*. If it satisfies *τ*, return to Step 8. Otherwise, return to Step 3.

 
*Step 8*. Then, it decodes the best individual, the clustering prototype *v*_*i*_ is calculated, the classification results of each sample are calculated, and this classification result is the clustering result of data set *X*.

## 5. MapReduce Framework

In order to improve the efficiency of modified immune evolutionary algorithm (MIEA) in processing large datasets, this paper designs the implementation scheme of MIEA in the MapReduce model. There are two main operations in the mechanism processing big data clustering tasks: updating the center of the class and fitness evaluation. Class center is updated based on MIEA. Fitness evaluation is to calculate the sum of Euclidean distance between each object and the center of mass and then find the global optimal value. The clustering program divides data objects into clusters, minimizes the sum of Euclidean distances between all objects and the center of mass, and takes it as the fitness function of MIEA. The data clustering process based on MIEA is shown in Figure 2.

## 6. Experiments and Analysis

In order to verify the performance of clustering and data mining in cloud computing environment, we conduct abundant experiments. Medical data are taken from http://archive.ics.uci.edu/ml/. The database is constantly updated. Donations of data are also accepted. The database type involves life, engineering, science, etc.; the record number is from several to hundred thousand pieces. The data selected in this paper are Breast Cancer Wisconsin (Original) Data Set. These data sets are from the clinical case reports of the university of Wisconsin hospital in the United States, and each data has 11 attributes.

Due to limited space, we display only few results in here. The computing platform is configured with Intel Core I7 4.0 GHz CPU, 16G Memory, and NVIDIA GTX 780 GPU. The algorithm is compiled by Apache Hadoop platform. The sampling frequency of big data is *f*_s_=20 kHz. The time center of big data clustering is *t*_0_=20 s. Size of the data is from 50 MB to 2 GB. Cross probability *p*_*c*_=0.95, variation probability *p*_*v*_=0.3, and fuzzy index *m*=2. We also select three state-of-the-art clustering methods to make comparisons including HGM [34], WPC [35], and ACCH [36].

### 6.1. Result 1

Table 1 is the description of 11 attributes of this dataset.

In this paper, the proposed algorithm is adopted to calculate the weight of each feature. Features with the weight less than a certain threshold will be removed. According to the actual situation in this paper, 2 and3 with the smallest weight will be removed. In the process of the algorithm, we will randomly select sample *R*. Different random numbers will lead to certain discrepancy in the weight of the result. Therefore, this paper adopts the average method by running it for 20 times. Then, we summarize the results to calculate the average value of each weight as shown in Figure 3.

By analyzing the data set, the importance of attribute weight can be obtained, which has some reference values for clinical diagnosis and can be used for the analysis of actual cases. This can avoid misdiagnosis as far as possible and improve the diagnosis speed and accuracy. According to the attributes, we obtain the object function optimal value as given in Table 2.

### 6.2. Result 2

To evaluate the performance of proposed algorithm, the composite data sets given in Table 3 are adopted. The four public data sets are assembled into a large data set, all of which are from UCI Machine Learning Repository with different attributes. Four data sets are randomly copied into several backups to form a large data set with 10^7^ records.

*F*-measure is adopted as the evaluation index of clustering quality. *F*-measure is calculated from two information indexes, precision, and recall rate, defined as

(16) $$\begin{array}{c} F\left(i,j\right)=\frac{2\cdot r\left(i,j\right)\cdot p\left(i,j\right)}{r\left(i,j\right)+p\left(i,j\right)}, \end{array}$$

where *j* represents the class generated by the cluster method, *i* denotes the class label of original dataset, and *r* and *p* represent recall rate and precision, respectively. Recall rate is defined as *r*(*i*, *j*)=*n*_*ij*_/*n*_*i*_. Precision is defined as *p*(*i*, *j*)=*n*_*ij*_/*n*_*j*_. Here, *n*_*ij*_ represents the divided class number of class *i*. *n*_*i*_ and *n*_*j*_ are the data sizes of class *i* and class *j*, respectively. For the data set with size *n*, the calculation formula of *F*-measure is

(17) $$\begin{array}{c} F=\underset{i}{\sum }\frac{n_{i}}{n}\underset{j}{\max}\left(F\left(i,j\right)\right), \end{array}$$

where the upper bound of *F* is 1. If the *F*-measure value is larger, then the clustering quality will be higher as shown in Table 4. With the increase of dataset number, the *F* value is slightly on the whole. However, the value of 0.817 of the proposed method is still higher than that of HGM, WPC, and ACCH.

The following experiments are for the feature extraction under cloud computation.

The original big data feature distribution is random as shown in Figure 4, and it is difficult to achieve feature extraction in the two-dimensional space regularity. We use the proposed algorithm for feature extraction and processing data clustering to build big data feature extraction model. The obtained feature extraction results are shown in Figure 5.

As can be seen in Figure 5, the proposed algorithm can effectively evaluate the feature extraction of big data in cloud computing; the beam focusing performance is good, which provides accurate basis for the data optimal clustering. Using different big data clustering optimization algorithms, we get the clustering center optimal performance curve as shown in Figure 6.

We also get the best value and mean value within 200 iterations as shown in Figures 7–10. And, we can know that the best value is with our proposed method.

## 7. Conclusions

In cloud computing environment, vast amounts of data need to be scheduled and accessed aiming at achieving the goal of medical data mining. This paper puts forward a new medical big data clustering algorithm based on modified immune algorithm. It firstly analyzes the big data structure model in the cloud computing environment to build big data feature extraction and information model. Designing immune optimization algorithm for clustering, it achieves the goal of optimization clustering for big data. Simulation results show that the proposed algorithm improves the clustering performance of big data in cloud computing environment. The new algorithm is used for IoT data clustering, which reduces the error rate and exhibits better performance. In the future, we will research the deep learning methods and apply them into actual engineering projects.

## Figures and Tables

**Figure 1:** Proposed clustering algorithm flow diagram.

**Figure 2:** Data clustering flow based on MIEA.

**Figure 3:** Weight change in 20 times.

**Figure 4:** Big data two-dimensional feature distribution in cloud computing.

**Figure 5:** Feature extraction result with the proposed method.

**Figure 6:** Comparison results.

**Figure 7:** HGM method.

**Figure 8:** WPC method.

**Figure 9:** ACCH method.

**Figure 10:** Proposed method.

**Table 1:** Attribute description.

Name of attributes	Description	The serial number of characteristics
Lumps thickness	1–10	1
Cell size uniformity	1–10	2
Cell morphology uniformity	1–10	3
Marginal adhesion	1–10	4
Single epithelial cell size	1–10	5
Bare nucleus	1–10	6
Bland chromatin	1–10	7
Normal nucleoli	1–10	8
Mitosis	1–10	9

**Table 2:** Performance comparison.

Method	HGM	WPC	ACCH	Proposed
Accuracy (%)	65	72	76	**85**
Optimal value	12.54	10.31	8.75	**6.59**

**Table 3:** Attributes of experimental datasets.

Number	Dataset	Sample number	Dimensionality	Cluster number
1	Iris	10000050	3	4
2	CMC	10000197	3	9
3	Wine	10000040	3	13
4	Vowel	10000822	6	3

**Table 4:** F comparison with different methods.

Dataset number	HGM	WPC	ACCH	Proposed
1	0.678	0.796	0.853	**0.912**
2	0.312	0.336	0.398	**0.423**
3	0.493	0.528	0.735	**0.796**
4	0.597	0.654	0.678	**0.817**

## Data Availability

The data used to support the findings of this study are available from the corresponding author upon request.
